# lncRNA MALAT1 Regulates Mouse Granulosa Cell Apoptosis and 17*β*-Estradiol Synthesis via Regulating miR-205/CREB1 Axis

**DOI:** 10.1155/2021/6671814

**Published:** 2021-02-17

**Authors:** Lei Sun, Pengju Zhang, Wenfa Lu

**Affiliations:** ^1^Joint Laboratory of Modern Agricultural Technology International Cooperation, Ministry of Education, Jilin Agricultural University, Changchun 130118, China; ^2^Institute of Animal Biotechnology, Jilin Academy of Agricultural Sciences, Changchan 130033, China

## Abstract

Metastasis-associated lung adenocarcinoma transcript 1 (MALAT1), a known long noncoding RNA, was reported to play a crucial role in follicular growth and ovarian disease. However, the physiological function of MALAT1 in mouse granulosa cells (mGCs) remains largely unclear. The aims of this study were to determine the biological function and molecular mechanism of MALAT1 in mGCs. We knocked down MALAT1 in mGCs by using siRNA against MALAT1. We found that knockdown of MALAT1 promoted apoptosis and caspase-3/9 activities in mGCs. Enzyme-linked immunosorbent assay demonstrated that knockdown of MALAT1 significantly decreased the production of estradiol (E2) and progesterone (P4) in mGCs. Mechanistically, MALAT1 serves as a competing endogenous RNA (ceRNA) to sponge microRNA-205 (miR-205), thereby facilitating its downstream target of cyclic AMP response element- (CRE-) binding protein 1 (CREB1). Furthermore, CREB1 overexpression or miR-205 downregulation partially recovered the effect of MALAT1 depletion in mGCs. In summary, these findings suggested that MALAT1 regulated apoptosis and estradiol synthesis of mGCs through the miR-205/CREB1 axis.

## 1. Introduction

It is well known that most ovarian follicles (>99%) in the mammalian ovary undergo atresia and degeneration, and only <1% of the follicles suffer ovulation [1, 2]. The high apoptosis ratio of GCs could impair folliculogenesis, leading to follicular atresia [3]. Especially, steroid hormones synthesized by GCs play an important role in ovarian follicular development, oocyte maturation, endometrial proliferation, and mammary gland development [4]. Therefore, exploring the molecular mechanism involved in GC progression is crucially important for decreasing follicular atresia and increasing ovulation rates and female fertility.

Long noncoding RNAs (lncRNAs) are a class of noncoding RNAs that are longer than 200 nucleotides in length and do not appear to have protein-coding potential [5]; they have been found to participate in various biological processes, such as early embryonic development [6], granulosa cell proliferation [7], and stem cell differentiation [8]. Moreover, some lncRNAs have been observed to be expressed in ovaries [9], mature and immature oocytes [10], and cumulus cells [11]. Growing evidence suggested that lncRNAs are involved in follicular growth and development through the regulation of GC proliferation, differentiation, apoptosis, and steroidogenesis [12–15]. Therefore, ovarian functional research related to lncRNAs was being performed extensively to clarify the molecular mechanism of follicular growth and development.

MALAT1, a key lncRNA, was reported to play pivotal roles in various malignancies, mainly by regulating the proliferation, migration, and invasion of cancer cells [16]. In the reproductive system, MALAT1 was shown to be associated with pregnancy loss [17], polycystic ovary syndrome (PCOS) [18], and endometriosis [19]. Although a study demonstrated that MALAT1 promoted human GC proliferation through the regulation of the ERK/MAPK pathway [20], the detailed function and regulatory mechanism of MALAT1 in mouse granulosa cells (mGCs) remain largely unclear. The present study is aimed at examining the potential involvement of MALAT1 in mGC proliferation, apoptosis, and estradiol synthesis. We also investigated the regulatory mechanism underlying the effect of MALAT1 on mGCs by conducting a series of molecular and cellular experiments *in vitro*.

## 2. Materials and Methods

### 2.1. Follicle Isolation

Follicles of C57BL/6j mouse were obtained from Dr. Wang (Jilin University). Based on the morphological characteristics of the follicles, they were divided into healthy follicles (HFs), early atretic follicles (EAFs), and progressively atretic follicles (PAFs).

### 2.2. mGC Culture and Transfection

Primary mGCs were isolated as described based on our previous study [21]. mGCs were grown in Dulbecco's modified Eagle's medium/nutrient mixture F-12 (DMEM/F12; Sigma-Aldrich, CA) supplemented with 10% inactivated fetal bovine serum (FBS; Gibco BRL, CA), penicillin (100 U/mL), and streptomycin (100 U/mL) (Life Technologies, CA) at 37°C in a humidified atmosphere with 5% CO_2_. The media were changed every 48 h. The 2- or 3-passage mGCs were selected for subsequent experiments.

A siRNA directly targeting MALAT1 (si-MALAT1; 5′-GTGAATGAGTGATAAGTAA-3′) and appropriate nontargeting siRNA (si-NC; 5′-TTCTCCGAACGTGTCACGT-3′) were bought from Geneseed Biotech Co. (Guangzhou, China). In addition, GenePharma Co. Ltd. (Shanghai, China) provided miR-205 mimics (5′-UCCUUCAUUCCACCGGAGUCUG-3′), negative control mimics (miR-NC; 5′-GGUCCGUCCGUAAUUAUCCUCC-3′), and a miR-205 inhibitor (anti-miR-205; 5′-CAGACUCCGGUGGAAUGAAGGA-3′) as well as its negative control (anti-miR-NC; 5′-CAGACUCCGGUGGAAUGAAGGA-3′). The CREB1 overexpression plasmid came from our lab. mGCs (5 × 10^3^ cells/well) underwent transient transfection with the abovementioned constructs (100 nM siRNAs, mimics and inhibitors) using Lipofectamine 3000 (Invitrogen, CA, USA) based on provided protocols, with the efficiency of transfection being assessed at 48 h following transfection by quantitative real-time PCR (qRT-PCR).

### 2.3. RNA Extraction and qRT-PCR

Total RNA was isolated from mGCs using the TRIzol Reagent (Invitrogen) according to the standard protocol. One *μ*g RNA was reverse transcribed to cDNA with the PrimeScript RT Reagent Kit (Takara Biotechnology Dalian Co. Ltd., Dalian, China). qRT-PCR was performed on an ABI Prism 7900 system (Applied Biosystems, CA, USA) using the SYBR Premix Ex Taq (Takara Biotechnology Dalian Co. Ltd., Dalian, China). The following thermocycling protocol was used: denaturation at 94°C for 5 min, followed by 40 cycles of denaturation at 94°C for 10 sec, annealing at 62°C for 20 sec, and extension at 72°C for 40 sec. The relative expression was calculated using the 2^−ΔΔCt^ method and normalized to GAPDH or U6. The sequences of primes are listed in Table 1 based on previous studies [22–24].

### 2.4. Apoptosis Assays

The apoptosis of mGCs was determined using Annexin V-FITC/PI apoptosis detection kits (A211, Vazyme, Nanjing, China) under fluorescence-activated cell sorting (FACS) following the manufacturer's protocols. The apoptotic rate of mGCs was calculated and analyzed using FlowJo software (v3.2, Stanford University, Stanford, CA, USA).

### 2.5. Caspase-3/9 Activity Assay

Caspase-3 Activity Assay Kit and Caspase-9 Activity Assay Kit (Beyotime, Beijing, China) were used to determine the activities of caspase-3/9 in mGCs 48 h after transfection according to the manufacturer's protocol. The OD value at 405 nm was measured using a microplate spectrophotometer (Thermo Labsystems, Vantaa, Finland).

### 2.6. Estradiol ELISA Assay

mGCs were harvested by centrifugation at 3000 × g for 5 min at 48 h. The concentrations of estradiol (E2) and progesterone (P4) were measured using the mouse estradiol (E2) ELISA kit (sensitivity: 2 ng/mL; cat. no. MU30395; Shanghai New Hualian Pharmaceutical Co., Ltd., Wuhan, China) and the mouse progesterone (P4) ELISA kit (sensitivity: 10 pg/mL; cat. no. WK-SU00650; Shanghai Walan Biotechnology Co., Ltd., Shanghai, China) based on the manufacturer's instructions, respectively.

### 2.7. Subcellular Fractionation Assay

The NE-PER Nuclear and Cytoplasmic Extraction Reagents (Thermo Fisher Scientific, Waltham, MA) were applied with the isolation of the nuclear and cytoplasmic extracts from mGC cells. The distribution of MALAT1 was determined in the cytoplasm or nucleus using qRT-PCR. GAPDH and U6 were used as cytoplasmic and nuclear controls, respectively.

### 2.8. Luciferase Reporter Assay

The miRNAs that interact with MALAT1 were predicted with starBase2.0 (http://starbase.sysu.edu.cn/). A dual-luciferase reporter gene assay was used to verify the target relationship between miR-205 and MALAT1. A wildtype (WT) or mutant-type (MT) MALAT1 fragment containing the miR-205 binding site was synthesized and inserted into the pGL3-basic vector (Promega, Madison, WI, USA). For luciferase reporter assay, 1 × 10^5^ mGCs were cotransfected with the WT-MALAT1 reporter plasmid and the MT-MALAT1 reporter plasmid and miR-205 mimics or miR-NC control. The luciferase reporter assay system (Promega) was applied to examine the luciferase activities at 48 h after cotransfection.

### 2.9. RNA Pull-Down Assay

1 × 10^4^ mGCs were transfected with biotinylated miR-205 wildtype (bio-miR-205-wt), miR-205 mutant type (bio-miR-205-mut), and negative control (bio-NC, GenePharma Co. Ltd., Shanghai, China), respectively). After 48 h of transfection, cell lysates were collected and incubated with M-280 streptavidin magnetic beads (Invitrogen, CA, USA) for 3 h at 4°C according to the manufacturer's protocol. Then, the beads were washed three times with ice-cold lysis buffer and once with high-salt buffer (Invitrogen). The bound RNAs were purified using TRIzol and then subjected to qRT-PCR to measure MALAT1 levels.

### 2.10. Western Blot Assay

The cultured mGCs were harvested and lysed using a radioimmunoprecipitation assay buffer (Sigma-Aldrich) according to the manufacturer's protocol. After the concentration was quantified with a bicinchoninic acid (BCA) kit (Sigma-Aldrich), an equal quantity of 30 *μ*g protein in each well was separated by 10% sodium dodecyl sulfate-polyacrylamide gel electrophoresis (SDS-PAGE) and then electrophoretically transferred onto a polyvinylidene difluoride (PVDF) membrane (Millipore, MA). After blocking with 5% nonfat milk for 1 h at room temperature, membranes were then incubated overnight at 4°C in the following primary antibodies: anti-CREB1 (1 : 500 dilution; cat. no: ab32515), anti-CYP19A1 (1 : 1000 dilution; cat. no: ab215443), anti-CYP1B1 (1 : 500 dilution; cat. no: ab185954), and anti-GAPDH (1 : 3000 dilution; ab8245). This was followed by incubation with a horseradish peroxidase-conjugated corresponding secondary antibody (1 : 5000 dilution; ab6721 or ab6789) at 37°C for 2 h. All of these antibodies were bought from Santa Cruz Biotechnology Inc. (Santa Cruz, CA). The protein signals were visualized using an enhanced chemiluminescence detection reagent on a Bio-Rad ChemiDoc MP system (Bio-Rad, Hercules, CA), and expression was normalized to GAPDH. Densitometry analysis of the gel images was conducted using the ImageJ software (v1.8.0; National Institutes of Health, Bethesda, MD, USA).

### 2.11. Statistical Methods

All the statistical data are shown as mean ± standard deviation (SD) of at least three independent experiments and three parallel holes in each experiment (*n* = 9). All statistical analyses were performed with SPSS 19.0 software (SPSS, Inc., Chicago, IL, USA). Student's *t*-test was used to compare differences between two groups, and multiple groups were compared with one-way ANOVA followed by Duncan's test as a post hoc test. *P* < 0.05 was taken into account as statistically significant.

## 3. Results

### 3.1. Knockdown of MALAT1 Promotes Apoptosis of mGCs

To investigate the expression of MALAT1 in follicles, we detected the expression levels of MALAT1 in HFs, EAFs, and PAFs by qRT-PCR. The results showed that the expression of MALAT1 in EAFs and PAFs were significantly lower than those in HFs (both *P* < 0.01; Figure 1(a)), suggesting that MALAT1 might be involved in follicular atresia. To further clarify the biological roles of MALAT1 in mGCs, the endogenous MALAT1 in primary mGCs was knocked down by siRNAs and the cell apoptosis and caspase-3/9 activities were determined by flow cytometry and ELISA, respectively. As shown in Figure 1(b), MALAT1 was successfully knocked down by 84.2% by si-MALAT1. Meanwhile, we found that knocking down MALAT1 significantly promoted the apoptotic cell number (Figure 1(c)) and increased caspase-3/9 activities (Figures 1(d) and 1(e)).

### 3.2. Knockdown of MALAT1 Decreases the Concentrations of Estradiol and Progesterone in mGCs

To assess whether MALAT1 affects steroid hormone levels in mGCs, we measured the concentrations of estradiol (E2) and progesterone (P4) in mGCs at 48 h postinfection by ELISA. The result revealed that the concentrations of E2 and P4 were significantly reduced in the si-MALAT1 group (both *P* < 0.01) compared with the si-NC group (Figures 2(a) and 2(b)). We further analyzed the expression of two genes encoding steroidogenic enzymes cytochrome P450 1B1 (CYP1B1) and CYP19A1 in mGCs transfected with si-MALAT1 or si-NC. The results revealed that MALAT1 depletion significantly reduced the CYP1B1 and CYP19A1 protein expression in mGCs (Figure 2(c)). These results suggest that MALAT1 might play a crucial role in the regulation of steroidogenesis in mGCs.

### 3.3. MALAT1 Is Targeted by miR-205

lncRNAs were reported to function as a competing endogenous RNA (ceRNA) by binding with miRNAs and regulating gene expression at the posttranscriptional level [25]. To determine the mechanism by which MALAT1 regulates mGC apoptosis, the miRNAs that directly interact with MALAT1 were predicted using the bioinformatics tool starBase2.0. Among the miRNAs, we select miR-205 as a study object based on its biological role in the reproduction field. MALAT1 harbors a recognition sequence of miR-205 (Figure 3(a)). This interaction was confirmed by dual-luciferase assay. As shown in Figure 3(b), overexpression of miR-205 significantly reduced the WT-MALAT1 luciferase activity of mGCs, but not that of MT-MALAT1. To further investigate the potential direct binding between MALAT1 and miR-205, RNA pull-down assays were performed in mGC cells, and this revealed that biotin-labeled miR-205-wt could pull down MALAT1, while bio-miR-205-mut could not pull down MALAT1 (Figure 3(c)), indicating the direct interaction between MALAT1 and miR-205. In addition, we found that knockdown of MALAT1 obviously increased miR-205 expression in mGCs (Figure 3(d)). We also showed that transfection of miR-205 mimics significantly increased miR-205 expression in mGCs, whereas transfection of the miR-205 inhibitor obviously decreased miR-205 expression in mGCs (Figure 3(e)). However, miR-205 upregulation or downregulation failed to cause alteration of MALAT1 expression in mGCs (Figure 3(f)). These results demonstrate that MALAT1 could bind to miR-205 in mGCs.

### 3.4. MALAT1 Exerts a Biological Role in mGCs by Regulating the miR-205/CREB1 Axis

A previous study demonstrated that miR-205 promoted mGC apoptosis by targeting CREB1 [23]. To investigate whether MALAT1 exerts a biological role in mGCs by modulating the miR-205/CREB1 axis, we first investigated the association with MALAT1, miR-205, and CREB1 in mGCs. We found that knockdown of MALAT1 significantly decreased CREB1 expression in mGCs, while transfection with the miR-205 inhibitor partially reversed this trend (Figures 4(a) and 4(b)). Finally, we found that downregulation of miR-205 or upregulation of CREB1 partially reversed the effect mediated by MALAT1 knockdown on proliferation, apoptosis, caspase-3/9 activities, and E2 and P4 production in mGCs (Figures 4(c)–4(g)). These results determine convincingly that MALAT1 exerts its biological function via the miR-205/CREB1 axis.

## 4. Discussion

Granulosa cells (GCs), a basic functional unit of the ovary, were reported to be involved in the growth and maturation of follicles by regulating proliferation, cell cycle, apoptosis, and synthesis of steroid hormones in female mammals [26]. Growing evidence indicates that the initiation of follicular atresia is mainly due to GC apoptosis [3, 22, 27]. Several lncRNAs have been identified as regulators of GC apoptosis in mammals. For example, the lncRNA NORFA inhibited granulosa cell apoptosis through regulating miR-126/transforming growth factor-*β* (TGF-*β*) axis [12]. Knockdown of PVT1 promoted cell proliferation, as well as inhibition of apoptosis of ovarian granulosa cells by regulating miR-17-5p and PTEN [28]. The lncRNA HOTAIR aggravated the endocrine disorders and granulosa cell apoptosis through competitive binding to miR-130a to upregulate the expression of IGF1 [14]. In this study, we prove that MALAT1 could affect apoptosis and estradiol synthesis of mGCs. We also demonstrate that MALAT1 plays an important role in regulating apoptosis and estradiol synthesis of mGCs through regulating the miR-205/CREB1 axis.

MALAT1, as a conserved lncRNA, was shown to be involved in multiple biological processes, such as tumorigenesis, pre-mRNA splicing, and DNA repair [16, 29, 30]. Although a study has revealed that MALAT1 might affect human GC proliferation through P21/P53-dependent control of the cell cycle and the ERK/MAPK pathway [20], the biological function of MALAT1 in follicular atresia remains largely unclear. In the present study, we observed MALAT1 reduction in EAFs and PAFs compared with HFs. Downregulation of MALAT1 decreased the centration of E2 and P4 in mGCs. We also showed that knockdown of MALAT1 significantly induced apoptosis and promoted caspase-3/9 activities in mGCs. These results suggested that MALAT1 might play a key role in follicular atresia.

Accumulating evidence suggested that dysregulated lncRNAs exert crucial regulatory functions in multiple processes through acting as ceRNAs to sponge microRNAs (miRNAs) [31]. MALAT1 was identified to sponge multiple miRNAs, such as miR-124-3p [32], miR-150-5p [33], miR-503 [34], miR-384 [35], and miR-22 [36]. To investigate the regulatory mechanism of MALAT1 in mGCs, we selected miRNA interactions with MALAT1 using starBase2.0 software. Among the miRNAs, we select miR-205 as a study object based on its biological function. Recently, a study demonstrated that miR-205 overexpression promoted apoptosis and decreased estradiol synthesis in mGCs [23]. Here, we confirmed that miR-205 could directly bind with MALAT1 in the luciferase reporter activity assay and RNA pull-down assays. We also found that knockdown of MALAT1 significantly increased miR-205 expression in mGCs, while overexpression or downregulation of MALAT1 did not alter the expression of MALAT1 in mGCs. In addition, miR-205 inhibition partially reversed the effect of MALAT1 depletion in mGCs. These results suggest that MALAT1 functions as a ceRNA by sponging miR-205 in mGCs.

Accumulating evidence confirmed that lncRNAs functioned as ceRNAs of miRNAs that cause the modulation of derepression of miRNA's target gene expression [25, 31]. CREB1 was confirmed to be a direct target of miR-205 in mGCs [23]. Importantly, knockdown of CREB1 could induce apoptosis and decrease the production of E2 and P4 in mGCs [37]. Thus, we investigate the association with CREB1, miR-205, and MALAT1 in mGCs. We found that knockdown of MALAT1 in mGCs resulted in a reduction in the expression of CREB1, while this trend was reversed by CREB1 overexpression. Moreover, MALAT1-mediated effects on apoptosis, caspase-3/9 activities, and E2 and P4 production were effectively rescued by CREB1 overexpression. These findings suggest that MALAT1 affects mGC apoptosis and estradiol synthesis via the miR-205/CREB1 axis.

In conclusion, the present study revealed that MALAT1 could regulate mGC apoptosis and steroid synthesis, at least to a certain extent by regulating miR-205/CREB1 axis. These findings contribute to an understanding of the molecular mechanisms underlying the regulation of ovarian follicular atresia by MALAT1.

## Figures and Tables

**Figure 1:** Knockdown of MALAT1 affects mGC proliferation and apoptosis. (a) The expression of MALAT1 in HFs, EAFs, and PAFs was determined using qRT-PCR. EAFs: early atretic follicles; HFs: healthy follicles; PAFs: progressively atretic follicles. (b) The expression of MALAT1 was examined in mGCs transfected with si-MALAT1 or si-NC. (c–e) Cell apoptosis and caspase-3/9 activities were determined in mGCs transfected with si-MALAT1 or si-NC. Data are the means ± SD (*n* = 3) of one representative experiment, ^∗^*P* < 0.05, ^∗∗^*P* < 0.01 vs. the HFs or si-NC group. mGCs: mouse granulosa cells; MALAT1: metastasis-associated lung adenocarcinoma transcript 1; qRT-PCR: quantitative RT-PCR.

**Figure 2:** Knockdown of MALAT1 decreases the concentrations of estradiol and progesterone in mGCs. (a, b) The E2 and P4 concentrations were measured in mGCs transfected with the si-NC or si-MALAT1. (c) The CYP1B1 and CYP19A1 protein expression levels were analyzed in mGCs transfected with si-NC or si-MALAT1. Data are the means ± SD (*n* = 3) of one representative experiment, ^∗^*P* < 0.05, ^∗∗^*P* < 0.01 vs. the si-NC group. mGCs: mouse granulosa cells; MALAT1: metastasis-associated lung adenocarcinoma transcript 1; CYP1B1: cytochrome P450 1B1; CYP19A1: cytochrome P450; family 19: subfamily a, polypeptide 1.

**Figure 3:** MALAT1 is targeted by miR-205 in mGCs. (a) The predicted miR-205 binding sites in the region of MALAT1 and the corresponding mutant sequences are shown. (b) Effect of miR-205 on the luciferase activity of WT-MALAT1 and MT-MALAT1 reporter systems was detected via luciferase reporter assay. (c) RNA pull-down assay was conducted to assess the relationship between miR-205 and MALAT1. (d) The expression of miR-205 was examined in mGCs transfected with si-MALAT1 or si-NC. (e) The expression of miR-205 was examined in mGCs transfected with miR-205 mimics, miR-NC, miR-205 inhibitor (anti-miR-205), and anti-miR-NC. (f) The expression of MALAT1 was examined in mGCs transfected with miR-205 mimics, miR-NC, miR-205 inhibitor (anti-miR-205), and anti-miR-NC. Data are the means ± SD (*n* = 3) of one representative experiment, ^∗^*P* < 0.05, ^∗∗^*P* < 0.01 vs. the si-NC group. mGCs: mouse granulosa cells; MALAT1: metastasis-associated lung adenocarcinoma transcript 1.

**Figure 4:** MALAT1 exerts a biological role in mGCs by regulating the miR-205/CREB1 axis. (a, b) The expression of CREB1 on mRNA and protein levels was examined in mGCs transfected with si-NC, si-MALAT, and si-MALAT1+anti-miR-205. (c–g) The apoptosis, caspase-3/9 activities, and E2 and P4 production were determined in mGCs transfected with si-NC, si-MALAT, si-MALAT1+anti-miR-205, and si-MALAT1+CREB1. Data are the means ± SD (*n* = 3) of one representative experiment, ^∗^*P* < 0.05, ^∗∗^*P* < 0.01 vs. the si-NC group. CREB1: encoding cyclic AMP response element- (CRE-) binding protein 1; mGCs: mouse granulosa cells; MALAT1: metastasis-associated lung adenocarcinoma transcript 1.

**Table 1:** Primer sequences for qRT-PCR analysis.

Target gene	Prime (5′-3′)
MALAT1	F-CCTAACGACTAGCATTGGCA
	R-GCACTCTTTCCTGGGCTATC
CREB1	F-AGCAGCTCATGCAACATCATC
	R-AGTCCTTACAGGAAGACTGAACT
GAPDH	F-TGTGTCCGTCGTGGATCTGA
	R-TGGCGGTGGCTCAGTTCAGC
miR-205	F-GTGCAGGGTCCGAGGT
	R-GATCCTTCATTCCACCGG
U6	F-CTCGCTTCGGCAGCACA
	R-AACGCTTCACGAATTTGCGT

Abbreviations: F = forward; mRNA = messenger RNA; PCR = polymerase chain reaction; R = reverse.

## Data Availability

The data from this study are available in this published article.
